The article "Clone Selection Artificial Intelligence Algorithm-Based Positron Emission Tomography-Computed Tomography Image Information Data Analysis for the Qualitative Diagnosis of Serous Cavity Effusion in Patients with Malignant Tumors" was published in 2021. Journal: J Healthc Eng.

# Clone Selection Artificial Intelligence Algorithm-Based Positron Emission Tomography-Computed Tomography Image Information Data Analysis for the Qualitative Diagnosis of Serous Cavity Effusion in Patients with Malignant Tumors

**DOI:** 10.1155/2021/4272411

**Published:** 2021-12-18

**Authors:** Jing Wei, Pingwei Li, Huai Zhang, Ronghua Zhu

**Affiliations:** ^1^Department of Nuclear Medicine, Huai'an First People's Hospital, 6 Beijing West Road, Huaiyin District, Huai'an 223300, Jiangsu, China; ^2^Department of Radiotherapy, Huai'an First People's Hospital, 6 Beijing West Road, Huaiyin District, Huai'an 223300, Jiangsu, China

## Abstract

This study aimed to investigate the application of positron emission tomography- (PET-) computed tomography (CT) image information data combined with serous cavity effusion based on clone selection artificial intelligence algorithm in the diagnosis of patients with malignant tumors. A total of 97 patients with PET-CT scanning and empirically confirmed as serous cavity effusion were retrospectively analyzed in this study. The clone selection artificial intelligence algorithm was applied to register the PET-CT images, and the patients were rolled into a benign effusion group and a malignant effusion group according to the benign and malignant conditions of the serous cavity effusion. Besides, the causes of patients from the two groups were analyzed, and there was a comparison of their physiological conditions. Subsequently, CT values of different KeV, lipid/water, water/iodine, and water/calcium concentrations were measured, and the differences of the above quantitative parameters between benign and malignant serous cavity effusion were compared, as well as the registration results of the clone algorithm. The results showed that the registration time and misalignment times of clonal selection algorithm (13.88, 0) were lower than those of genetic algorithm (18.72, 8). There were marked differences in CT values of 40–60 keV and 130–140 keV between the two groups. The concentrations of lipid/water, water/iodine, and water/calcium in basal substances of the malignant effusion group were obviously higher than the concentrations of the benign effusion group (*P* < 0.05). Benign and malignant effusions presented different manifestations in PET-CT, which was conducive to the further diagnosis of malignant tumors. Based on clone selection artificial intelligence algorithm, PET-CT could provide a new multiparameter method for the identification of benign and malignant serous cavity effusions and benign and malignant tumors.

## 1. Introduction

Serous cavity effusion (SCE) is a common symptom and sign in clinical work, which is divided into pleural effusion, ascites, and pericardial effusion [1, 2]. When the effusions occur in two or more parts of the patient's body simultaneously or successively during the course of the disease, they are called polyserositis. The causes of SCE are often complicated, and the common causes include malignant tumor, tuberculosis, hypoproteinemia, and hepatogenic, nephrogenic, cardiogenic, and autoimmune diseases [3–5]. At present, there are various methods for detection of SCE. The frequently used methods contain biochemical examination, tumor marker, exfoliated cell detection, flow cytometry, and telomerase activity assay. However, the detection rates of these methods are generally low, so it is often necessary to carry out repeated tests to get more accurate results [6]. Moreover, the traditional imaging detections such as X-ray, ultrasound, and computed tomography (CT) can only detect diseases by relying on morphological changes, and it is impossible to achieve more effective inspections for early disease [7, 8]. At this stage, medical diagnosis and treatment capabilities with the further advancement of E-health have been improved directly or indirectly from digital medical equipment to high-level information and knowledge sharing, and various digital imaging and postprocessing technologies make disease diagnosis more intuitive and accurate. Under this background, positron emission tomography- (PET-) CT has gradually been applied in the detection of SCE. The PET-CT imaging is a method combining molecular metabolism with anatomical structure images. It has obvious advantages in early identification and diagnosis of most diseases [9]. The detection method is easy to operate and noninvasive and lets patients suffer little pain. After long-term clinical application, it has been proved to have obvious advantages in the differential diagnosis of various diseases. Above all, it has been applied better in identifying the nature of effusion and finding the primary lesion of malignant effusion [10, 11]. In addition, the registration based on the shape feature points of the PET-CT image is difficult and requires the application of external reference point features for registration. However, due to the characteristics of mutual information function and multiple extreme values, there are usually multiple local extreme values, so that the optimization process may converge to the local extreme value and get wrong registration parameters, resulting in mismatching of image registration. In recent years, clonal selection algorithm is widely used in pattern recognition and combinatorial optimization. Its core is to multiply replication operator and mutation operator, retain the best individual, and improve the poor individual. It is an efficient and fast convergence algorithm. Therefore, the patients were detected by PET-CT using clone selection artificial intelligence algorithm in this study, and patients with benign and malignant effusions were evaluated, thereby providing new ideas for clinical treatment of peripheral facial paralysis and pointing out new directions.

The article "Clone Selection Artificial Intelligence Algorithm-Based Positron Emission Tomography-Computed Tomography Image Information Data Analysis for the Qualitative Diagnosis of Serous Cavity Effusion in Patients with Malignant Tumors" was published in 2021. Journal: J Healthc Eng.

## 2. Methods

### 2.1. Subjects Investigated and Grouping

97 patients who underwent PET-CT scanning in hospital from June in 2017 to June 2019 and were empirically diagnosed as SCE were retrospectively analyzed. In the patients with malignant effusion, the primary lesions of some with malignant tumors have been confirmed by pathology, except for others with liver cirrhosis and primary liver cancer. According to the nature of effusion, 97 patients were divided into benign and malignant effusion, including 25 benign and 72 malignant. All the patients participating in the experiment had signed informed consent forms, and this study had been approved by ethics committee of hospital.

### 2.2. Inclusion and Exclusion Criteria

The inclusion criteria for the patients participating in the experiment were as follows: the patients met the diagnostic criteria of Western medicine, were above 20 years and below 65 years of age, had no other acute diseases or severe complications during the period of developing SCE, and were under no other treatment.

The exclusion criteria of patients participating in the experiment were as follows: patients in pregnancy or early pregnancy, having severe cardiovascular and cerebrovascular diseases, liver and kidney function disease, and hematopoietic failure, having cerebral infarction, cerebral hemorrhage, or other brain diseases, having participated in other clinical experiments, not developing SCE for the first time, and having the disease again after receiving treatments on the first onset.

### 2.3. Immunohistochemical Staining Reaction

The SCE was made into a smear and rinsed; after that, the smear was soaked in the permeable solution for 5 minutes, and then phosphate buffer solution (PBS) was applied to rinse the soaked smear. The rinsed section was added with PBS to be incubated in an incubator at 37°C for 30 minutes. After the incubation, the enzyme reaction solution was added to the incubated section for light avoidance reaction, and it was rinsed after 1 hour of the light avoidance reaction. Then, fluorescein isothiocyanate (FITC) working solution was added to continue the reaction for 30 minutes in the dark; and the section was rinsed after the reaction finished. Finally, 4′,6-diamidino-2-phenylindole (DAPI) working solution was dropped on the surface of the section, which was observed with a computer fluorescence microscope.

The article "Clone Selection Artificial Intelligence Algorithm-Based Positron Emission Tomography-Computed Tomography Image Information Data Analysis for the Qualitative Diagnosis of Serous Cavity Effusion in Patients with Malignant Tumors" was published in 2021. Journal: J Healthc Eng.

### 2.4. Positron Emission Tomography-Computed Tomography Scanning Detection Method

The Discovery ST 4 PET-CT instrument was for PET-CT scanning, and Advanced PET and Lightspeed 4-slice spiral computed tomography (CT) were combined on the same machine rack. Before the detection, the patient should fast for 4–6 hours in advance, and the fasting blood glucose of the patient had to be less than 7 mmol/L. If the patient's blood glucose was too high before the detection, the insulin should be injected appropriately to control the blood glucose within the normal range. After the patient stayed at rest for 15 minutes, the patient was given an intravenous injection of imaging agent with the amount of 3.71–4.82 MBq/kg. After the injection, the patient would continue to maintain a resting state for 45–60 minutes. Moreover, PET-CT scanning was applied immediately after the patient urinated. During the detection, the patient was placed in a supine position, held his head with his hands, kept breathing calm, and was scanned from the top of the skull to the upper femur on both sides. Gemstone spectral imaging (GSI) mode was used for CT scanning, with a spiral scanning speed of 0.6 s/ week, a detector width of 4 cm, a voltage of instantaneous switching between high and low energy (140 kVp and 80 kVp), and a tube current of about 600 mA. The first group of image reconstruction was the common 140 kVp image, which was used for real-time observation during the detection process, with a layer thickness/layer interval of 5 mm. The second group was a single energy (70 keV) image with a layer thickness/layer interval of 1.25 mm. In addition, standard algorithms were employed for image reconstruction.

### 2.5. PET-CT Image Registration Based on Clone Selection Algorithm

The clone selection process is a positive feedback process, and the clone selection algorithm is employed to find the maximum value of normalized mutual information and its corresponding registration parameters. The specific steps are as follows.

The first step is initialization. The PET-CT image is used as the initial research object, corresponding to the possible solutions of registration parameters. The floating-point number is encoded, and the base number is 19, in which the first 10 bits correspond to the rotation parameters of the image space transformation, and the last 9 bits correspond to the scale parameters of the image transformation. The probability of crossover is set as *Yi* = 0.7 and the probability of mutation as *Yt* = 0.02. The second step is evaluation and selection. The normalized mutual information value is calculated; the larger 30 of them are selected to enter the memory set Pn and the remaining Pm. The third step is clone. In the memory set Pn, K with higher normalized mutual information value are selected for cloning, and the number of clones is proportional to the fitness. It is ensured that the selection of registration parameters develops towards the optimization direction.

The article "Clone Selection Artificial Intelligence Algorithm-Based Positron Emission Tomography-Computed Tomography Image Information Data Analysis for the Qualitative Diagnosis of Serous Cavity Effusion in Patients with Malignant Tumors" was published in 2021. Journal: J Healthc Eng.

The fourth step is crossover and mutation. The supermutation process in biological clone selection is simulated, and the cross-mutation operation is carried out on the results after clone, so the mutation rate is inversely proportional to the fitness, thus enlarging the search range of registration parameters. The fifth step is the second evaluation and selection. The affinity of the mutated antibodies is recalculated. If the affinity of some clone results is higher than that of the highest Pn, the body with the lowest affinity in Pn is replaced with these antibodies to form a new memory set. The sixth step is extinction. The process of natural cell extinction in biological clonal selection is simulated. In Pm, *d* results with the lowest affinity are selected to reinitialize, which can ensure the speed of convergence. The seventh step is to check whether the termination conditions are met. If they are met, terminate; otherwise, go to the second step and enter the next generation avoidance.

The clone algorithm can realize the diversity of the search space and optimize the objective function of medical image registration, with good performance.

### 2.6. Image Processing, Analysis, and Measurement

The image analysis and measurement were on the professional workstation AW4.5. Three radiologists with ten years of work experience carried out the measurement independently, and they did not know the final results of the subjects investigated. On the mixed energy 140 kVp imaging image, the most obvious layer of the effusion in the image was selected to measure the CT value. Besides, circular reactive oxygen intermediate (ROI) with a diameter of 5–10 mm was selected, and three-point measurement was carried out, and the average value was selected. The single energy image (70 keV, and 5 mm) was loaded into spectrum imaging analysis software GSI viewer for analysis. The ROI of the same patient was measured against the corresponding region of the mixed energy, and the ROI data file was saved. The data file was an Excel spreadsheet file, containing the CT value (HU) of each single energy level 40–140 keV (the interval for 10 keV) and effective atomic number; the statistical software was employed to calculate the peak of effective atomic number distribution; and lipid (water), water (iodine), and water (calcium) were selected as the paired base substances, and their concentrations were generated by the data file.

The article "Clone Selection Artificial Intelligence Algorithm-Based Positron Emission Tomography-Computed Tomography Image Information Data Analysis for the Qualitative Diagnosis of Serous Cavity Effusion in Patients with Malignant Tumors" was published in 2021. Journal: J Healthc Eng.

### 2.7. Statistical Analysis

SPSS 17.0 statistical analysis software was used for the statistical methods. The results of counting were expressed as mean ± standard deviation ($\bar{x}$ ± *s*), and *t*-test was applied for comparison between the two groups. The receiver operating characteristic curve (ROC) was employed to evaluate the value of paired base substances in the diagnosis of malignant effusion, and AUC was applied to determine the accuracy of base substance concentration in the diagnosis of malignant effusion. What is more, the threshold value, sensitivity, and specificity for the diagnosis of malignant effusion were calculated, and *P* < 0.05 was considered to represent statistically significant difference.

## 3. Results

### 3.1. Comparison of the Basic Data of Patients

Based on the nature of the effusion, 97 patients were classified into benign and malignant effusion, respectively. There were 25 patients with benign effusion including 11 males and 14 females, the average age was 62.17 ± 6.33 years, and the course of disease was 2.57 ± 0.24 years. What is more, 72 patients were malignant effusion including 33 males and 39 females, with an average age of 63.74 ± 4.76 years and the disease course of 3.57 ± 1.24 years. The results in Figure 1 show that the difference in general data between the two groups of patients was not statistically remarkably significant (*P* > 0.05).

### 3.2. Analysis of the Causes of the Patients in the Two Groups

There were 25 patients in the benign effusion group, and their specific causes are shown in Figure 2. The benign effusion group included 8 patients of liver cirrhosis with ascites, 2 patients of heart failure with pleural effusion, 13 patients of pneumonia with pleural effusion, and 2 patients of tuberculous pneumonitis with ascites.  Figure 3 shows the specific causes of 72 patients in the malignant effusion group. Besides, there were 14 patients of gastrointestinal malignant tumors with ascites, 44 patients of lung cancer with pleural effusion, 9 patients of breast cancer with multiple metastases and pleural effusion, 3 patients of ovarian cancer with ascites, and 2 patients of esophageal cancer with pleural effusion in the malignant effusion group. There was no statistical difference in the number of cases of each cause of the above patients (*P* > 0.05).

### 3.3. Comparison of the Physiological Conditions of the Patients in the Two Groups

The two groups of patients were subjected to immunohistochemical tests, and the representative results were selected for display shown in Figure 4. In addition, the immunohistochemical results of the benign effusion group showed that there was a small amount of positive cells; namely, the overall degree of cell malignancy was not high; meanwhile the immunohistochemical results of the malignant effusion group indicated that the positive cells were abundant in the effusion; namely, the whole cells had the high degree of malignancy.

The article "Clone Selection Artificial Intelligence Algorithm-Based Positron Emission Tomography-Computed Tomography Image Information Data Analysis for the Qualitative Diagnosis of Serous Cavity Effusion in Patients with Malignant Tumors" was published in 2021. Journal: J Healthc Eng.

### 3.4. Comparison of PET-CT Image Registration Values between Clone Selection Algorithm and Genetic Algorithm

Figure 5 discloses that the average difference of the maximum value of the normalized mutual information of PET-CT image registration of the clone selection algorithm is small, with no statistically huge difference (*P* > 0.05). Furthermore, the registration time and mismatching times were lower than those of genetic algorithm, and the differences were statistically substantial (*P* < 0.05).

The lungs were further taken as the comparison objects. The pneumonia with pleural effusion and lung cancer with pleural effusion were selected as the examples of the benign and malignant effusion group, respectively, as shown in Figure 6. In the PET-CT image of benign effusion, it is shown that there were concentrated shadows of radioactive distribution in lymph nodes and the larger range of lesion, so that they were presumed to be infectious lesions, and pneumonia was diagnosed based on medical history. There was no obvious radioactive concentrated area in the PET-CT image of malignant effusion, so as to speculate to be lung cancer with lymph node metastasis and diagnose lung cancer combined with medical history.

### 3.5. The CT Values of the Patients in the Two Groups under Different Energies

The differences in CT of the patients from the two groups were compared under different energies, and the results are expressed in Figure 7. Under the low energy (40–60 keV), the CT values of the benign effusion group were 41.24 ± 18.45 HU, 31.75 ± 12.8 HU, and 25.78 ± 11.12 HU; and the CT values of the malignant effusion group were 0.96 ± 19.45 HU, 7.99 ± 12.48 HU, and 12.57 ± 11.22 HU, with a statistical difference between the two groups (*P* < 0.05). Under 70–120 keV, the CT values of the benign effusion group were 21.15 ± 6.27 HU, 18.11 ± 6.33HU, 15.99 ± 5.24 HU, 15.24 ± 8.45 HU, 15.02 ± 4.21 HU, and 14.71 ± 6.66 HU; the CT values of malignant effusion group were 15.82 ± 7.67 HU, 17.55 ± 10.63 HU, 19.33 ± 11.27 HU, 20.01 ± 9.67 HU, 20.14 ± 10.44 HU, and 21.98 ± 10.57 HU, and the difference between the two groups was not statistically dramatic (*P* > 0.05). Under 130–140 keV, the CT values of the benign effusion group were 14.11 ± 6.17 HU and 13.56 ± 6.54 HU, while the CT values of the malignant effusion group were 21.44 ± 11.66 HU and 21.97 ± 12.57 HU; thus, there was a statistical difference in the two groups (*P* < 0.05).

The article "Clone Selection Artificial Intelligence Algorithm-Based Positron Emission Tomography-Computed Tomography Image Information Data Analysis for the Qualitative Diagnosis of Serous Cavity Effusion in Patients with Malignant Tumors" was published in 2021. Journal: J Healthc Eng.

### 3.6. The Paired Base Substances of the Patients in the Two Groups

Figure 8 illustrates that the contents of lipid/water, water/iodine, and water/calcium in malignant effusion were sharply higher than the contents of benign effusion. What is more, the content of lipid/water in malignant effusion was 221.44 ± 189.45 g/L, while its content in the benign effusion was 201.45 ± 197.56 g/L; the contents of water/iodine in the malignant and benign effusion were 1024.69 ± 19.48 g/L and 1008.48 ± 18.27 g/L, respectively; and the contents of water/calcium in the malignant and benign effusion were 1027.87 ± 11.66 g/L and 1009.48 ± 9.21 g/L, respectively. Therefore, there was a statistical difference between the two groups (*P* < 0.05).

Figure 9 demonstrates that the diagnostic sensitivity, specificity, and AUC of malignant effusion were 95.5%, 92.6%, and 97.7%, respectively, when the lipid/water concentration was over 104.34 g/L; when the water/iodine concentration was more than 1024.22 g/L, the diagnostic sensitivity, specificity, and AUC of malignant effusion were 86.4%, 77.8%, and 79.8%, respectively; and the diagnostic sensitivity, specificity, and AUC of malignant effusion were 86.4%, 92.6%, and 86.7%, respectively, when the water/calcium concentration was greater than 1028.44 g/L.

## 4. Discussion

Serous cavity refers to the human chest, abdominal cavity, pericardial cavity, and so forth. Under normal conditions, only a small amount of fluid in the serous cavity provides lubrication and protection (the fluid in the pleural cavity <20 mL, the fluid in the peritoneal cavity <50 mL, and the fluid in the pericardial cavity 10–50 mL). However, the increased volume of fluid in the cavity leads to the occurrence of effusion under pathological conditions, which is called SCE. Once the disease is complicated by SCE, it often indicates the severity of the disease [12, 13]. Based on the causes of the effusion, the effusion can be divided into benign and malignant. The study of Sherman-Samis et al. (2019) showed that many common causes of benign SCE were decompensation of liver cirrhosis, cardiac insufficiency, renal function failure, tuberculosis, and nonspecific inflammation. However, malignant SCE often existed in the late stages of various malignant tumors. This was because the blood vessels and lymph vessels were invaded by malignant tumor, or lymph nodes metastasis was to hinder the backflow and absorption of SCE; or tumor cells directly invaded blood vessels to increase the capillary permeability [14]. It was consistent with the pathological detection results of the study. The gold standard for diagnosing malignant effusion is to find tumor cells in SCE, but only when the malignant tumor invades the pleura or peritoneum or directly falls off in the effusion will a positive result be obtained. Moreover, its specificity is high, but the positive rate is low [15]. Das proved in a study that 58% was the positive rate of a single test in the pleural effusion. In addition, there was a false negative rate in the detection of malignant exfoliative cytology, and its sensitivity was only 40–60% [16]. Therefore, the PET-CT scanning detection proposed in the experiment plays an important role in assisting the diagnosis of malignant effusion. It has great advantages in the diagnosis of tumors, and it can diagnose most tumors on the double-layer structure and functional metabolism through whole body imaging. What is more, it has very critical significance in finding the primary tumor lesion, and the nature diagnosis of patients with pleural and abdominal effusion is also relatively clear [17–19].

The article "Clone Selection Artificial Intelligence Algorithm-Based Positron Emission Tomography-Computed Tomography Image Information Data Analysis for the Qualitative Diagnosis of Serous Cavity Effusion in Patients with Malignant Tumors" was published in 2021. Journal: J Healthc Eng.

Harrison et al. summarized and sorted out the diseases that produced serous cavity effusion. The results illustrated that the main cause was malignant tumors in the chest and abdominal cavity, and pericardial effusion and tuberculosis also accounted for a large proportion, followed by connective tissue diseases, inflammatory infection, liver cirrhosis, heart function failure, hypothyroidism, and nephrotic syndrome [20]. The results were similar to the results of the study. However, there are certain differences in details, which may be caused by too few samples in the study. The PET-CT imaging based on the artificial intelligence algorithm of clone selection injects a small amount of positron nuclide tracer into the human body. The commonly used tracer is PF-FDG, which is adopted to detect the distribution of these positron nuclides in various organs of the human body. CT is employed to display the physiological metabolism of the main organs of the human body and to accurately locate, thereby fusing images. In this study, the clone selection algorithm was used to find that the registration time and mismatching times were both low, which achieved the optimal registration of PET-CT images and improved the accuracy of imaging results [21–23]. Zaucha et al. [24] stated that PET-CT was of great significance in finding primary tumor lesions and was more accurate in the diagnosis of patients with pleural and ascites effusion. It was also consistent with the experimental results of the study, showing that it is more sensitive to the diagnosis of malignant tumors. The paired base substances of lipid (water), water (iodine), and water (calcium) contents were selected for analysis, because the range of substances commonly used in medicine from fat to iodine contrast agents was included [25]. Knorr et al. have proved that free fatty acids in malignant ascites were 3 times higher than those in liver cirrhosis, and both saturated and unsaturated fatty acids in malignant ascites were higher than those in liver cirrhosis [26]. This is because fatty acids are the energy substrate for tumor cell metabolism, and malignant effusion contains dense and abundant tumor cells, which grow and metabolize vigorously, so lipids increase in malignant ascites [27–30]. It was reflected in the results of the study, indicating that the liquid concentration of the malignant effusion was higher than that of the benign effusion.

The article "Clone Selection Artificial Intelligence Algorithm-Based Positron Emission Tomography-Computed Tomography Image Information Data Analysis for the Qualitative Diagnosis of Serous Cavity Effusion in Patients with Malignant Tumors" was published in 2021. Journal: J Healthc Eng.

## 5. Conclusion

In this study, there was an investigation on the effect of PET-CT imaging detection image information and data information based on clone selection artificial intelligence algorithm in the diagnosis of serous cavity effusion in patients with different types of tumors. Besides, it was analyzed according to benign effusion and malignant effusion. It was found that the registration time and the times of mismatching of PET-CT images under the clone selection algorithm were both low, and the optimal registration of PET-CT images was realized. The image results indicated that benign and malignant serous cavity effusion could not be distinguished by CT values of routine mixed energy and 70–80 keV single energy (equivalent to mixed energy), while the CT value of low energy (40–60 keV) image played a critical role in the identification of benign and malignant effusions. However, the overall sample size of this study is small, and only relevant analysis for benign effusion and malignant effusion does not analyze many other clinical factors and the prognosis of patients. In the future, the sample size will be expanded to conduct more in-depth and comprehensive research and exploration in this direction. In short, PET-CT based on the artificial intelligence algorithm of clone selection has important diagnostic value in unexplained serous cavity effusion and has high sensitivity, specificity, and accuracy in the diagnosis of malignant pleural effusion.

## Figures and Tables

**Figure 1:** Comparison of the basic data of the patients in the two groups. (a) Comparison of the gender among the patients in the two groups; (b) comparison of the age and course of disease among the patients in the two groups.

**Figure 2:** The disease causes of the patients with benign effusion.

The article "Clone Selection Artificial Intelligence Algorithm-Based Positron Emission Tomography-Computed Tomography Image Information Data Analysis for the Qualitative Diagnosis of Serous Cavity Effusion in Patients with Malignant Tumors" was published in 2021. Journal: J Healthc Eng.

**Figure 3:** The disease causes of the patients with malignant effusion.

**Figure 4:** The immunohistochemical results of the patients in the two groups. (a) The results of benign effusion group; (b) the results of malignant effusion group.

**Figure 5:** PET-CT image registration values. Note. (a) The average value of the maximum normalized mutual information; (b) registration time; (c) the times of mismatching. ^*∗*^ indicates that the difference compared with clone selection algorithm is statistically significant.

**Figure 6:** The PET-CT images of two patients. (a) PET-CT image of the pneumonia with pleural effusion patient; (b) PET-CT image of the lung cancer with pleural effusion patient.

**Figure 7:** The CT values of benign and malignant effusion under different energies.

**Figure 8:** Comparison of the concentrations of paired base substances in the benign and malignant effusion.

**Figure 9:** The ROC curve of paired base substances for diagnosis of malignant effusion.

## Data Availability

The data used to support the findings of this study are available from the corresponding author upon request.
